# COMTVal158Met Genotype Affects Complex Emotion Recognition in Healthy Men and Women

**DOI:** 10.3389/fnins.2018.01007

**Published:** 2019-01-22

**Authors:** Alexander Lischke, Rike Pahnke, Jörg König, Georg Homuth, Alfons O. Hamm, Julia Wendt

**Affiliations:** ^1^Department of Psychology, University of Greifswald, Greifswald, Germany; ^2^Institute of Sport Sciences, University of Rostock, Rostock, Germany; ^3^Interfaculty Institute for Genetics and Functional Genomics, University Medicine Greifswald, University of Greifswald, Greifswald, Germany

**Keywords:** COMT, catecholamine, 5-HTTLPR, serotonin, emotion recognition, social cognition

## Abstract

The catechol-o-methyltransferase (COMT) gene has repeatedly been shown to change amygdala activity and amygdala-prefrontal connectivity during face processing. Although the COMT gene appears to induce a negativity bias during the neural processing of faces, it is currently unclear whether a similar negativity bias emerges during the behavioral processing of faces. To address this issue, we investigated differences in complex emotion recognition between participants (*n* = 181) that had been *a priori* genotyped for functional polymorphisms of the COMT (Val158Met) and serotonin transporter (5-HTTLPR) gene. We were, thus, able to analyze differences in face processing on basis of participants’ COMT genotype while controlling for participants’ 5-HTTLPR genotype. Variations of participants’ COMT but not 5-HTTLPR genotype accounted for differences in participants’ emotion recognition performance: Met/Met carriers and Met/Val carriers were more accurate in the recognition of negative, but not neutral or positive, expressions than Val/Val carriers. We, therefore, revealed a similar negativity bias during the behavioral processing of faces that has already been demonstrated during the neural processing of faces, indicating that genotype-dependent changes in catecholamine metabolism may affect face processing on the behavioral and neural level.

## Introduction

Over the last two decades, there has been a growing interest to determine the genetic basis of social behavior (Ebstein et al., 2010). Social behavior crucially depends on the processing of facial cues providing information about others’ intentions, thoughts and emotions. Consequently, much research has been devoted to delineate the genetic mechanisms underlying face processing (Niedenthal and Brauer, 2012). However, most research dealt with these mechanisms on the neural not behavioral level, presumably because neural processes are more susceptible to genetic variations than behavioral processes (Hariri and Weinberger, 2003). As a result, we know a lot about the genetic modulation of neural activity during face processing, but almost nothing about the behavioral consequences of this genetic modulation.

Of the various genes implicated in face processing, the catechol-o-methyltransferase (COMT) gene appears to be of particular relevance (Montag et al., 2012). The COMT gene regulates the extracellular degradation of catecholamines (dopamine, norepinephrine, and epinephrine). A single nucleotide polymorphism predicts the substitution of amino acid methionine (Met) for valine (Val) at codon 158 (VAL158MET), which results in a threefold to fourfold reduction of catecholamine degradation in Met as compared to Val carriers (Lachman et al., 1996). The associated differences in extracellular catecholamine levels appear to account for neural differences in face processing as suggested by imaging studies revealing increased amygdala activity (Williams et al., 2010; Lonsdorf et al., 2011) and increased amygdala-prefrontal connectivity (Surguladze et al., 2012) in response to negative expressions in Met carriers. Met carriers, thus, show an enhanced processing of negative expressions, indicating a negativity bias during face processing. However, such a negativity bias has not always been found in behavioral studies (Weiss et al., 2007; Defrancesco et al., 2011; Gohier et al., 2014). Two studies failed to find robust differences in emotion recognition between Met and Val carriers (Weiss et al., 2007; Defrancesco et al., 2011), whereas a third study revealed that Met carriers misperceived neutral expressions as negative ones (Gohier et al., 2014). Met carriers may, thus, not only show an enhanced processing of negative expressions as suggested by the imaging studies (Williams et al., 2010; Lonsdorf et al., 2011; Surguladze et al., 2012) but also a negatively tuned processing of neutral expression as suggested by one of the behavioral studies (Gohier et al., 2014). In this respect, it is important to note that this behavioral study (Gohier et al., 2014) differed markedly from the other two behavioral studies (Weiss et al., 2007; Defrancesco et al., 2011) in terms of sample size (e.g., inclusion of more than 100 participants), genotype frequencies (e.g., consideration of COMT and 5-HTTLPR polymorphisms), task design (e.g., presentation of expressions with varying emotional intensity) and data analysis (e.g., control of multiple comparisons). Methodological differences between the behavioral studies may, thus, have accounted for the inconsistent findings regarding Met carriers negativity bias during face processing. Consequently, there is a need for studies that investigate differences in emotion recognition between Met and Val carriers with more methodological rigor.

In the present study, we further investigated whether Met and Val carriers differ in emotion recognition. In contrast to previous studies (Weiss et al., 2007; Defrancesco et al., 2011; Gohier et al., 2014), we employed a task that required the recognition of complex rather than basic emotional expressions (Reading the Mind in the Eyes Test, RMET; Baron-Cohen et al., 2001). We decided to use complex expressions for our task because these expressions resemble more the type of expressions one encounters throughout social interactions than basic expressions (Zelenski and Larsen, 2000). The set of complex expressions is also much larger than the set of basic expressions (Cordaro et al., 2018), which usually comprises six different expressions (Ekman et al., 1969). Due to the large number of different expressions, our task was far more challenging than the tasks that had been employed in previous studies (Weiss et al., 2007; Defrancesco et al., 2011). We, thus, expected to detect subtle differences in emotion recognition, which may have not been the case in previous studies (Weiss et al., 2007; Defrancesco et al., 2011). The task was administered to a sample of participants that had been *a priori* genotyped for functional polymorphisms of the COMT and serotonin transporter (5-HTTLPR) gene. We *simultaneously* considered participants’ COMT and 5-HTTLPR genotype in our analyses because some studies suggest that the 5-HTTLPR genotype also affects face processing (Lonsdorf et al., 2011; Surguladze et al., 2012; Gohier et al., 2014). These analyses were based on an *a priori* power analysis and corrected for multiple comparisons to guard of false positive or false negative findings, indicating that our analyses were liberal and conservative enough to detect meaningful differences in face processing. As the aforementioned studies suggest that the negativity bias in face processing is more pronounced in Met than Val carriers (Williams et al., 2010; Lonsdorf et al., 2011; Surguladze et al., 2012; Gohier et al., 2014), we expected Met carriers to recognize more negative expressions than Val carriers.

## Materials and Methods

### Participants

Previous studies investigated how the COMT genotype modulated face processing in young to middle-aged participants of European descent (Weiss et al., 2007; Williams et al., 2010; Defrancesco et al., 2011; Lonsdorf et al., 2011; Surguladze et al., 2012; Gohier et al., 2014). We, thus, decided to include participants with an European background and an age range of 18–40 years in our study. Although none of the participants appeared to be of Asian descent, we did not formally check whether participants were indeed Caucasians. As the emotion recognition task required a fluent understanding of German, we excluded participants from the study whose native language was not German. In order to estimate the minimum number of participants that we needed to detect differences in emotion recognition on basis of participants’ COMT and 5-HTTLPR genotype, we performed an *a priori* power analysis with the freely available program G^∗^Power (Faul et al., 2007). Of note, as we were only interested in genotype- not allel-dependent differences in emotion processing, we solely based our power analysis on participants’ genotype. G^∗^Power indicated that we had to recruit at least 144 participants to have sufficient power (1-β = 0.80, α = 0.05) to detect medium-sized differences in emotion recognition (*f* = 0.25) in a multi-factorial analysis of variance (ANOVA) with the within-subjects factor expression valence and the between-subjects factors genotype. Allowing for attrition, we recruited 181 participants from a database of healthy volunteers who had been *a priori* genotyped for functional polymorphisms of the COMT and 5-HTTLPR gene (Wendt et al., 2015). All participants provided written-informed consent for the study protocol, which was approved by the ethics committee of the University of Greifswald and carried out in accordance with the Declaration of Helsinki.

### Genotyping

Details regarding the genotyping procedure can be found elsewhere (Wendt et al., 2015). In brief, standard procedures were used to extract DNA from whole blood (Autopure LS System, Gentra Systems, Minneapolis, MN, United States), a 5′-exonuclease TaqMan^®^ assay (C_25746809; Applied Biosystems, Foster City, CA, United States) was used for genotyping of the COMT VAL158MET (rs4680) polymorphism and polymerase chain reaction primers (forward 5′-TGAATGCCAGCACCTAACCCCTAA-3′, reverse 5′-GAATACTGGTAGGGTGCAAGGAGA-3; Thermo Scientific, Ulm, Germany) were used for genotyping of the triallelic 5-HTTLPR (5-HTTLPR/rs255331) polymorphism. Genotyping of the COMT VAL158MET polymorphism resulted in 54 Met/Met, 86 Met/Val and 41 Val/Val carriers, while genotyping of 5-HTTPLPR polymorphism resulted in 44 s/s, 85 s/l, and 52 l/l carriers. The distribution of the different COMT and 5-HTTLPR genotypes is illustrated in Tables 1, 2.

**Table 1:** Genotype distribution.

	COMT VAL158MET		
	Met/Met carriers	Met/Val carriers	Val/Val carriers
5-HTTLPR	*N*	*N*	*N*
s/s carriers	16	22	6
s/l carriers	23	36	26
l/l carriers	15	28	9


**Table 2:** Participant characteristics.

	Sex (m/f)	Age (years)		Psychopathology (BSI-18-GSI)	
	*N*	*M*	*SEM*	*M*	*SEM*
**COMT VAL158MET**					
Met/Met carriers	25/29	26.28	0.44	0.35	0.38
Met/Val carriers	47/39	26.18	0.35	0.27	0.28
Val/Val carriers	24/17	27.84	0.60	0.26	0.22
**5-HTTLPR**					
s/s carriers	23/21	26.18	0.56	0.26	0.27
s/l carriers	41/44	27.03	0.35	0.30	0.29
l/l carriers	32/20	27.10	0.49	0.29	0.26


*m, male; f, female; BSI-18-GSI, brief symptom inventory 18 global severity index (Franke et al., 2017)*.

### Psychopathology

The Brief Symptom inventory (BSI-18; Franke et al., 2017) was used to asses participants’ psychopathological distress at the time of the study. The BSI-18, which measures anxious, depressive and somatoform symptoms within the last 7 days, demonstrated good psychometric properties [BSI-18: α = 0.82].

### Emotion Recognition

A computerized version of the Reading the Mind in the Eyes Test (RMET; Baron-Cohen et al., 2001) was used to assess participants’ emotion recognition abilities. Whereas other emotion recognition tasks, like, for example, the morphed emotion recognition test (Lischke et al., 2012), required the recognition of basic emotional expressions (e.g., fear or happiness), the RMET required the recognition of complex emotional expressions (e.g., contempt or pride). The complex expressions had to be recognized on basis of subtle cues that were provided by the eye region of faces. These eye regions were randomly presented in form of 37 different black and white pictures (1 picture was used for practice and 36 pictures were used for testing). Each eye region was shown together with four labels describing distinct emotional expressions (see Figure 1). One label described the depicted emotional expression (target label), whereas three other labels described emotional expressions that did not correspond to the depicted emotional expression (distractor labels). Participants had to select the label that best described the emotional expression by pressing a corresponding button as fast as possible. Similar as in previous studies (Hysek et al., 2012; Lischke et al., 2017; Pahnke et al., 2018), an established algorithm was used to determine the percentage of correctly identified positive, negative and neutral expressions on basis of participants’ responses (Harkness et al., 1999).

**FIGURE 1:** Example of a black and white picture that was used in the Reading the Mind in the Eyes test (Baron-Cohen et al., 2001). The picture shows an eye region and labels that describe four different expressions (one target label, three distractor labels). Participants had to identify the label that correctly described the depicted expression (panicked).

### Statistical Analysis

SPSS 22 (SPSS Inc., Chicago, IL, United States) was used for all analyses. Chi-square tests and 3 × 3 ANOVAs (COMT genotype × 5-HTTLPR genotype) were run to investigate genotype dependent differences in participants’ age, sex and psychopathology. A 3 × 3 × 3 ANOVA (COMT genotype × 5-HTTLPR genotype × Expression Valence) was run to investigate genotype dependent differences in participants’ emotion recognition. The significance level for all analyses was set at *p* ≤ 0.05 (two-sided) and, if appropriate, corrected for multiple comparisons using the Bonferroni method (Shaffer, 1995). Partial eta squared ($\eta_{p}^{2}$ ) was reported as an effect size measure to facilitate the interpretation of significant findings (Cohen, 1988).

## Results

### Participant Characteristics

Chi-square tests revealed a comparable proportion of participants with differences in 5-HTTLPR genotype among participants with differences in COMT genotype [χ^2^ (*N* = 81, *df* = 4) = 6.436, *p* = 0.169]. There were also no differences in the proportion of male and female participants across participants with different COMT or 5-HTTLPR genotypes as indicated by another series of chi-square tests [all χ^2^ ≤ 2.306, all *p* ≥ 0.316]. A 3 × 3 ANOVA (COMT genotype × 5-HTTLPR genotype) suggested age differences among participants with different COMT but not 5-HTTLPR genotypes [effect of COMT genotype: *F*(2,172) = 3.065, *p* = 0.049, $\eta_{p}^{2}$ = 0.034; all other effects and interactions involving 5-HTTLPR genotype and COMT genotype: all *F* ≤ 1.249, all *p* ≥ 0.292, all $\eta_{p}^{2}$ ≤ 0.028]. *Post hoc* tests showed that Met/Met and Met/Val carriers were of same age [*p* = 1.000] but of younger age than Val/Val carriers [*p* = 0.111 and *p* = 0.052, respectively]. Consequently, age was used as a covariate in the subsequent analyses. A 3 × 3 ANCOVA (COMT genotype × 5-HTTLPR genotype) revealed no differences in psychopathological distress among participants with different COMT or 5-HTTLPR genotypes [all effects involving COMT genotype, 5-HTTLPR genotype or the interaction of COMT and 5-HTTLPR genotype: all *F* ≤ 2.210, all *p* ≥ 0.113, all $\eta_{p}^{2}$ ≤ 0.025]. Of note, psychopathological distress was generally very low among participants with different COMT or 5-HTTLPR genotypes, indicating that participants were in good mental health at the time of the study. Table 2 provides an overview about the aforementioned participant characteristics.

### Emotion Recognition

A 3 × 3 × 3 ANCOVA (COMT genotype × 5-HTTLPR genotype × Expression Valence) indicated valence dependent differences in emotion recognition among participants with different COMT but not 5-HTTLPR genotypes [effect of COMT genotype: *F*(2,171) = 3.361, *p* = 0.037, $\eta_{p}^{2}$ = 0.038; interaction of COMT genotype and expression valence: *F*(3.62,309.30) = 3.124, *p* = 0.019, $\eta_{p}^{2}$ = 0.035; all other effects and interactions involving COMT genotype, 5-HTTLPR genotype or expression valence: all *F* ≤ 1.80, all *p* ≥ 0.085, all $\eta_{p}^{2}$ ≤ 0.040]. Follow-up 3 × 3 ANCOVAs (COMT genotype × 5-HTTLPR genotype) revealed that these differences emerged during the processing of negative [effect of COMT genotype: *F*(2,171) = 6.378, *p* = 0.002, $\eta_{p}^{2}$ = 0.069; all other effects and interactions involving COMT genotype or 5-HTTLPR genotype: all *F* ≤ 0.906, all *p* ≥ 0.462, all $\eta_{p}^{2}$ ≤ 0.021], but not positive [all effects and interactions involving COMT genotype or 5-HTTLPR genotype: all *F* ≤ 1.972, all *p* ≥ 0.101, all $\eta_{p}^{2}$ ≤ 0.044] or neutral [all effects and interactions involving COMT genotype or 5-HTTLPR genotype: all *F* ≤ 1.020, all *p* ≥ 0.363, all $\eta_{p}^{2}$ ≤ 0.012] expressions. *Post hoc* tests indicated that Met/Met and Met/Val carriers, who did not differ from one another [*p* = 0.722], were more accurate in the recognition of negative expressions than Val/Val carriers [*p* = 0.002 and *p* = 0.015, respectively]. Figure 2 demonstrates the aforementioned differences in emotion recognition on basis of participants’ COMT genotype.

**FIGURE 2:** Barplots showing differences in complex emotion recognition as a function of COMT genotype. Met/Met and Met/Val carriers were more accurate in the recognition of negative expressions than Val/Val carriers. Bars represent M +/– SEM. ^∗^*p* ≤ 0.05; ^∗∗^*p* ≤ 0.001.

## Discussion

Across a series of well-powered and comparison-corrected analyses, we were able to demonstrate that differences in participants’ COMT but not 5-HTTLPR genotype accounted for differences in participants’ emotion recognition performance. Met/Met and Met/Val carriers were more accurate in the recognition of negative, but not positive or neutral, expressions than Val/Val carriers, indicating a negativity bias in face processing. Of note, studies that failed to reveal a negativity bias in face processing in Met carriers did not simultaneously consider differences in participants’ COMT and 5-HTTLPR genotype in their analyses (Weiss et al., 2007; Defrancesco et al., 2011). Moreover, these analyses were neither well-powered nor comparison-corrected (Weiss et al., 2007; Defrancesco et al., 2011), implying the possibility of false positive or false negative findings. The findings of these studies should, thus, be treated with caution (Weiss et al., 2007; Defrancesco et al., 2011). Another study, however, simultaneously considered variations of the COMT and 5-HTTLPR genotype in their well-powered and comparison-corrected analyses (Gohier et al., 2014). This study revealed a negativity bias in face processing among Met carriers (Gohier et al., 2014), indicating that the failure to detect such a bias in the other studies may have been due to the aforementioned methodological limitations (Weiss et al., 2007; Defrancesco et al., 2011). Give that our study shared many methodological similarities with this study, it appears plausible to assume that Met carriers show increased recognition biases and recognition accuracies for negative expressions on the behavioral level. This assumption is also compatible with other studies that revealed an increased processing of negative expressions on the neural level in Met carriers. Notably, Met carriers showed an increase in amygdala activity (Williams et al., 2010; Lonsdorf et al., 2011) and amygdala-prefrontal connectivity (Surguladze et al., 2012) in response to basic expressions of negative valence. As the amygdala is also implicated in the recognition of complex expressions (Baron-Cohen et al., 1999; Adolphs et al., 2002), similar activity and connectivity changes may have occurred while Met carriers were processing complex expressions of negative valence. Moreover, the amygdala is highly susceptible to catecholamine transmission (Hariri et al., 2002; Onur et al., 2009), implying that genotype dependent changes in catecholamine metabolism may in fact account for Met carriers’ negativity bias during face processing.

It should be noted, however, that several genes are implicated in the catecholamine metabolism via enzyme activity and/or receptor density. Polymorphisms of the dopamine beta-hydroxylase gene, for example, also account for changes in catecholamine metabolism that are associated with differences in face processing (Gong et al., 2014). Moreover, face processing is also modulated by genes that change metabolisms of other neurotransmitters than catecholamine ones. Polymorphisms of the oxytocin receptor gene, for instance, are associated with differences in face processing via changes in oxytocin metabolism (Rodrigues et al., 2009). It, thus, seems likely that multiple genes, either alone or in concert, modulated participants’ face processing in the present study. Given the complexity of genetic influences on face processing, it may be too simplistic to assume that differences in participants’ face processing were solely due to differences in participants’ COMT genotype.

Consequently, it has to be determined in future studies whether catecholamine induced changes in amygdala activity and amygdala-prefrontal connectivity in fact account for the negativity bias in face processing that has been observed in Met as compared to Val carriers (Williams et al., 2010; Lonsdorf et al., 2011; Surguladze et al., 2012; Gohier et al., 2014). Notwithstanding that the neurobiological mechanisms underlying this negativity bias remain unclear, it seems plausible to assume that Met carriers perceive their social interactions as more negative than Val carriers because of this negativity bias. As a consequence, Met carriers may be more vulnerable to negative experiences in social interactions. These negative experiences may lead to anxious and depressive feelings, which may eventually manifest themselves in anxious and depressive symptoms or disorders. This may explain why Met carriers experience more anxiety and depression related symptoms or disorders than Val carriers (Montag et al., 2012). It may, thus, be interesting to investigate in longitudinal studies whether Met and Val carriers’ performance on face processing tasks is differentially associated with Met and Val carriers’ risk to develop anxiety or depression related disorders. Ideally, these studies should comprise large number of participants that have been genotyped for polymorphisms of multiple genes that have been shown to be associated with face processing on the neural and behavioral level. These studies may help to determine whether genotype dependent differences in face processing represent biomarkers with utility for the development of interventions that are concerned with the prevention or treatment of anxiety and depression related disorders. We hope that findings of the present study, which have to be replicated and extended, stimulates this type of research.

## Author Contributions

AL and JW designed the study. JK and JW collected the data. AL, GH, and RP analyzed the data. AL and RP wrote the manuscript. AH, GH, JK, JW, and RP contributed to writing, reviewing, and editing of the manuscript. All authors approved the final version of the manuscript.

## Conflict of Interest Statement

The authors declare that the research was conducted in the absence of any commercial or financial relationships that could be construed as a potential conflict of interest.
